The article "Risk of Hepatobiliary-Gastrointestinal Malignancies and Appropriate Cancer Surveillance in Patients With Primary Sclerosing Cholangitis" was published in 2021. Journal: Cureus.

# Risk of Hepatobiliary-Gastrointestinal Malignancies and Appropriate Cancer Surveillance in Patients With Primary Sclerosing Cholangitis

**DOI:** 10.7759/cureus.19922

**Published:** 2021-11-26

**Authors:** Sujani Yadlapati, Thomas A Judge

**Affiliations:** 1 Gastroenterology and Hepatology, Cooper University Hospital, Camden, USA; 2 Gastroenterology, Cooper University Hospital, Camden, USA

**Keywords:** cancer surveillance, hepatobiliary tumours, ibd associated cancer, cholangiocarcinoma, primary sclerosing cholangitis

## Abstract

Patients with primary sclerosing cholangitis (PSC) are at risk of hepatobiliary and gastrointestinal cancers. Increased risk of cancer is a result of the chronic, progressive fibro-inflammatory state which ultimately results in the destruction of biliary ducts. PSC is often associated with inflammatory bowel disease (IBD). Patients with PSC are at significant risk of cholangiocarcinoma (CCA), gall bladder malignancy and those with IBD are at increased risk of colorectal cancer. It is important to implement cancer surveillance protocols in these patients. The aim of these protocols is the prevention or early detection of cancerous or pre-cancerous lesions. Given that PSC is rare, large prospective studies evaluating the risk of malignancy in these patients are not available. A great deal of uncertainty exists regarding how to best implement cancer surveillance in these patients. About 50% of deaths in PSC patients are due to malignancy and many patients eventually progress to end-stage liver disease and succumb to hepatic failure. In this review, we cover cancer surveillance strategies in PSC patients based on existing literature and expert opinions.

## Introduction and background

Primary sclerosing cholangitis (PSC) is characterized by chronic hepatobiliary inflammation that causes stricturing disease in the biliary tree. Prevalence of PSC within the United States (US) is 4 to 15 per 100,000 people [1,2]. PSC has been observed in the American and European populations and less commonly in black and Asian populations [3]. With progressive biliary fibrosis, these patients progress towards end-stage liver disease and liver failure. Life expectancy from the time of diagnosis has been reported to be as short as 9 years and as long as 20 years [4]. About 5% of IBD patients develop PSC and close to two-thirds of PSC patients have IBD. Chronic inflammation increases the risk of gastrointestinal malignancies. Patients with PSC are at high risk of hepatobiliary cancers and patients with both PSC and IBD (PSC-IBD) also have an elevated risk of colon cancer compared to patients with IBD alone [5].

Malignancy is a major cause of mortality in PSC patients. These patients have up to 40 times higher risk of developing hepatobiliary cancer [6]. Malignancies associated with PSC include cholangiocarcinoma (CCA), colorectal cancer, gallbladder adenocarcinoma and hepatocellular carcinoma (HCC) [7]. In this review, we aim to discuss epidemiology and surveillance strategies utilized in the prevention and early detection of these malignancies. Although there is a lack of validated protocols for cancer surveillance, we review available diagnostic modalities for screening based on existing evidence and expert opinion.

## Review

Cholangiocarcinoma in PSC

Cholangiocarcinoma (CCA) has up to six-fold more in PSC-IBD patients compared to the general population [8]. Incidence as high as 24.2 out of 100,000 cases has been described [9]. There is a two-fold higher risk of CCA in patients with UC than those with Crohn’s disease (CD) [10]. CCA often occurs at a younger age in this population. PSC is often regarded as a transitional step in the development of CCA [10,11]. Ten-year risk of developing CCA in patients with PSC is about 9% [5]. CCA carries a critical prognosis with survival rates less than 10% at five years [12]. Predictors for the development of CCA among PSC patients have not been clearly established. Smoking, advanced age, alcohol use, duration of IBD, prior proctocolectomy, evidence of colon cancer or dysplasia at PSC diagnosis and polymorphism of the NKG2D gene are some previously mentioned risk factors for CCA. This evidence is yet to be validated [7,13]. 

At present, there are no standardized screening protocols for early recognition of CCA. Chronic inflammation in PSC results in biliary ductal changes. These changes can obscure early CCA recognition. PSC can involve either distal or central bile ducts, also referred to as small or large duct involvement. PSC involving larger intra-hepatic ducts and the biliary confluence is at accelerated risk of cancerous transformation compared to distal or smaller duct disease.

Societal guidelines published by the American Association for the Study of Liver Diseases (AASLD) and American College of Gastroenterology (ACG), advise a combination of imaging, such as ultrasound or MRI with magnetic resonance cholangio-pancreatography (MRCP), and tumor markers, such as carbohydrate antigen 19-9 (CA 19-9). biannually for CCA surveillance [14,15]. In contrast, the European Association for Study of Liver Disease (EASL) does not recommend any one particular imaging or biochemical marker in the detection of CCA [16]. Endoscopic retrograde cholangio-pancreatography (ERCP) with brush cytology sampling has also been described as an important diagnostic test in CCA detection but its precise role in screening protocols has not been defined. 

A reasonable method to screening is periodic imaging of biliary tree with MRI/MRCP or ultrasound. In contrast to computerized tomography (CT), both these imaging modalities have limited contrast and radiation exposure, making them more suitable screening modalities. Characteristic radiologic findings include distinctive signal enhancement and the presence of a mass. MRI/MRCP is more sensitive for the detection of early CCA compared to ultrasound. MRCP, when used as sole imaging modality, has a sensitivity of 78% and specificity of 76% in the detection of CCA [15]. MRCP in conjunction with MRI increases sensitivity to 89%. While the specificity of ultrasound in the detection of CCA is as high as 94%, reported sensitivity tends to be lower compared to MRCP [15].

CA 19-9 is currently the only available biomarker for CCA screening. CA 19-9 value more than or equal to 20 U/mL augments MRI/MRCP sensitivity to 100% but lowers specificity (38%) and accuracy (47%) in screening [17]. A CA 19-9 value exceeding 129 U/mL or more enhances the specificity but diminishes the sensitivity [17]. About one-third of the patients who meet this cut-off value do not have CCA. Small percentage of the general population has negative Lewis antigen and therefore would not benefit from CA 19-9 testing [18]. ERCP with brush cytology in combination with CA 19-9 above 20 U/mL is 100% sensitive with an accuracy of 49% for detection of CCA [15]. Positive ERCP findings include stenosis of bile ducts with polypoid duct lesion, strictures, or distinct proximal bile duct dilation [17]. ERCP with cytology lacks sensitivity in the detection of CCA. Bile duct brushing is often specific (84%-89%) but lacks sensitivity (8-100%) and therefore is a poor screening tool [17]. Fluorescence in situ hybridization (FISH) analysis from bile duct brushings is used to detect chromosomal irregularities. This increases the sensitivity and specificity of typical cytology [19,20]. A notable risk of ERCP is pancreatitis. Other risks are that of standard endoscopy such as bleeding, infection, and perforation. Patients undergoing ERCP should be carefully selected given invasive nature of this procedure.

Gallbladder malignancy in PSC

Primary sclerosing cholangitis patients are at an increased risk of gall bladder malignancy. Lifetime risk of developing gall bladder cancer in these patients is about 2% [21]. Several studies have looked at gall bladder pathology in PSC patients undergoing cholecystectomy. In a study by Said and colleagues 286 patients were screened for gall bladder pathology. Gall bladder masses were found in 6% of patients and pathology from cholecystectomy revealed that more than half of these cases were adenocarcinoma [22]. In another American study similar results were observed. Over 50% of patients who had cholecystectomy for gall bladder mass or polyp had adenocarcinoma [23]. Based on available data, current guidelines recommend cholecystectomy in PSC patients with gall bladder polyps greater than 8 mm [15]. Gall bladder masses of any size are considered high risk and these patients should undergo cholecystectomy [16]. Smaller polyps may be closely monitored. Cholecystectomy should be performed only in cases where the benefits of undergoing surgery outweigh risks. PSC patients are considered high risk for surgery. Therefore, prophylactic cholecystectomy in the absence of symptoms or clear indications should not be pursued. Five-year survival among patients with gall bladder malignancy is 5-10%. These patients should undergo right upper quadrant ultrasound at least once a year.

Hepatocellular carcinoma in PSC

There is limited data on the incidence of HCC in patients with PSC. Lifetime incidence of less than 3% has been reported by various studies [24]. Currently, gastrointestinal societies (AASLD, EASL, ACG) recommend HCC surveillance in those with PSC-related cirrhosis. These patients should have HCC surveillance imaging every 6 months. In the absence of cirrhosis, surveillance of HCC is often accomplished indirectly at the time of CCA and gall bladder cancer surveillance.

Colon cancer in patients with PSC-IBD

The majority of PSC patients have IBD, particularly ulcerative colitis subtype. Patients who have both PSC and IBD are at a higher risk of colon cancer compared to those with PSC or IBD alone. Several studies have revealed up to four-fold increase in the risk of CRC in patients with concurrent UC and PSC [25]. Previously published literature also suggests that PSC-IBD patients genotypically vary compared to IBD patients without PSC. These patients often develop colorectal cancer at a younger age, have rapidly progressive clinical course, develop more extensive colitis with increased frequency of right-sided cancers and overall have poor prognosis unlike typical IBD patients [26]. Increase in risk of CRC after liver transplantation has also been reported in prior literature [26]. Colonoscopy with biopsies is recommended in these patients at the time of PSC diagnosis. Colonoscopy should be repeated at 1-2-year intervals [14,16]. For patients with PSC alone, in the absence of IBD, some experts recommend colonoscopy at 3-5-year intervals [14,16]. It is unclear if use of chromoendoscopy with targeted biopsies is superior to high-definition colonoscopy in these cases. Many experts reserve chromoendoscopy for cases with particularly elevated CRC risk such as those with significant family history of colon cancer, PSC-IBD and extensive longstanding colitis. Risk of CRC remains undiminished in PSC-IBD patient’s post-transplant. Screening should be continued in these patients to reduce the risk of CRC. 

Pancreatic cancer in PSC

There is conflicting data on whether PSC is truly associated with increased risk of pancreatic cancer. One study reported by Bergquist, and colleagues noted a risk of pancreatic cancer up to 14 times higher in PSC patients than in the general population [7]. However, subsequent studies based in Netherlands and Belgium found a negligible risk of pancreatic malignancy in these patients [5,27]. Given lack of sufficient data, screening for pancreatic cancer is not recommended in patients with PSC.

A brief summary of surveillance strategies along with lifetime risk are listed in Table 1. Early treatment is imperative in these patients (Figure 1). Treatment strategies although briefly mentioned here are not discussed in its entirety in this article.

**Table 1:** Summary of risk and cancer screening recommendations in patients with primary sclerosing cholangitis. CCA: cholangiocarcinoma; HCC: hepatocellular carcinoma; PSC: primary sclerosing cholangitis; MRI: magnetic resonance imaging; MRCP: magnetic resonance cholangio-pancreatography; US: ultrasound.

Malignancy	Risk	Screening strategy
CCA	10% at 10 years [28]	Ultrasound or MRI/MRCP with CA 19-9 every 6-12 months [15]
Gallbladder cancer	2% lifetime incidence [21]	Annual ultrasound [14-16]
Colon cancer	PSC and IBD: Up to 15% and 30% risk at 10 and 20 years [5] 10x risk over general population [29] 4x more than UC patients [29]	PSC-IBD patients should undergo yearly colonoscopy. Chromo-endoscopy should be use if available [14,15]. PSC alone – colonoscopy every 3-5 years [15]
HCC	Less than 3% [30]	Not recommended. Yearly US to assess for Gall bladder malignancy inadvertently addresses HCC. Biannual US in those with cirrhosis
Pancreatic cancer	Insufficient evidence	Not recommended

**Figure 1:** Overview of follow-up and treatment strategies in PSC patients undergoing cancer screening. PSC: primary sclerosing cholangitis; CCA: cholangiocarcinoma; CRC: colorectal cancer; MRI: magnetic resonance imaging; MRCP: magnetic resonance cholangio-pancreatography; US: ultrasound; LGD: low-grade dysplasia; HGD: high-grade dysplasia.

## Conclusions

The goal of cancer surveillance in PSC is to diagnose cancer in asymptomatic patients in the hope that early identification will improve outcomes. CCA is associated with high mortality and early detection can significantly aid with improved survival. In this review, we covered the prevalence of various hepatobiliary/GI malignancies in PSC and screening strategies. While the treatment of these malignancies is not addressed in this article, a summary of treatment approaches is depicted. Currently, we need larger prospective and retrospective studies to truly determine cancer incidence in these patients, and to determine appropriate timing for surveillance. Based on available data, a reasonable approach to screening is the use of ultrasound or MRI/MRCP along with CA 19-9 every 6-12 months. At this time there are no standardized guidelines for screening in these patients; however, based on available data an effort should be made to improve cancer detection in this high-risk population. Patients with dominant stricture on imaging should then undergo ERCP with brushings and FISH if available. Those with PSC-IBD should undergo annual colonoscopy. Chromoendoscopy should be used if available. Yearly ultrasound should be done to screen for gall bladder malignancy. Screening for HCC in the absence of cirrhosis and pancreatic cancer is not recommended at this time however can be pursued for diagnostic purposes if additional risk factors are present. 
